RETRACTED

# IFC-305 attenuates renal ischemia-reperfusion injury by promoting the production of hydrogen sulfide (H_2_S) via suppressing the promoter methylation of cystathionine γ-lyase (CSE)

**DOI:** 10.1080/21655979.2022.2062105

**Published:** 2022-05-13

**Authors:** Jie Jiang, Chuling Wen, Yi Li, Guohui Liu, Zijun Chen, Dongwen Zheng

**Affiliations:** Nephrology Department, Dongguan People’s Hospital Affiliated to Southern Medical University, Dongguan, China

**Keywords:** Renal I/R, homocysteine, CSE, H_2_S, oxidative stress, IFC-305

## Abstract

Renal ischemia-reperfusion (I/R) injury is characterized by elevated expression of homocysteine and decreased production of hydrogen sulfide (H_2_S). Cystathionine γ-lyase (CSE) is a key factor in the onset of renal I/R injury, while IFC-305 can regulate the expression of CSE via epigenetic modification. Animal and cellular models of I/R were established in this work, followed by H&E staining to evaluate the extent of renal tissue injury under distinct conditions. Several methods, including ELISA, qPCR and Western blot, were used to analyze the levels of creatinine, CSE and H_2_S in various I/R models. Bisulfite sequencing PCR was used to evaluate the level of DNA methylation. The severity of the renal injury was significantly elevated in I/R rats and alleviated by the IFC-305 treatment. The level of Hcy was increased in the renal tissue and peripheral blood of I/R rats, while the IFC-305 treatment inhibited the expression of homocysteine (Hcy). Mechanistically, the DNA methylation in the CSE promoter was dramatically enhanced in I/R rats and cells, while the IFC-305 treatment reduced the level of DNA methylation in the CSE promoter. Moreover, the IFC-305 increased the concentration of H_2_S, which was reduced in I/R rats and cells. Finally, I/R rats and cells showed aberrantly high levels of MDA and superoxide, while the IFC-305 treatment reduced the levels of malondialdehyde (MDA) and superoxide. IFC-305, an adenosine derivative, promoted the production of H_2_S and attenuated renal injury in cellular and animal models of renal I/R by modifying the methylation status of the CSE promoter.

## Highlights

- IFC-305 treatment prevented I/R induced kidney injury.
- Hcy is up-regulated and CSE is down-regulation of CSE in I/R rats.
- IFC-305 restored the DNA methylation status of the CSE promoter in I/R rats.
- IFC-305 restored the levels of H2S, MDA and superoxide in I/R rats.
- IFC-305 increased the activity of CSE in HK-2 cells.
- IFC-305 restored the levels of H2S, MDA and superoxide in the Hcy-treated HK2 cells.

## Introduction

The ischemia-reperfusion (I/R) of the kidney can lead to acute renal injuries featured by a high rate of mortality. So far, there are no treatments or drugs with the ability to completely cure I/R injuries [1]. I/R injuries can be caused by a wide range of factors, such as abnormal levels of chemokine cytokines and reactive oxygen species (ROS) [1,2]. For example, ROS plays a major role in the induction of renal I/R injuries because ROS can induce the peroxidation of lipids, the dysfunction of proteins, the disruption of cytoskeletal structures, the degradation of cell-matrix, and the induction of immune reactions [1,3,4]. A wide range of agents has been proved to provide protection during treatment in I/R injuries in various animal models [5]. And some results obtained even suggested the possibility for further investigations with clinical trials. However, for most agents investigated, the effectiveness of a certain agent is still questioned over the long-term clinical use of some of the negative results published.

RETRACTED

H_2_S plays an essential role as a gasotransmitter and neuromodulator to participate in the regulation of a wide range of physiological activities [6,7]. H_2_S is generated from cysteine and homocysteine under the action of multiple synthases such as cysteine aminotransferase, 3-mercaptopyruvate sulfurtransferase, cystathionine γ-lyase (CSE), and cystathionine β-synthase (CBS) [8]. Among them, CBS can regulate the conversion of Hcy into cystathionine, which can then be converted to L-cysteine and α-ketobutyrate under the action of CSE. Finally, the metabolism of L-cysteine produces H_2_S. It was demonstrated previously that the inhibition of H_2_S synthesis could reduce the levels of CSE and CBS expression. It was also demonstrated that Hcy can repress the transcription of CSE in macrophages via enhancing the level of DNA hypermethylation in the promoter of CSE, subsequently reducing the synthesis of H_2_S and elevating the generation of certain cytokines in macrophages to promote inflammatory reactions. Moreover, Hcy increases the level of DNMT activity and expression. In summary, the above findings suggested that the inhibition in the synthesis of CSE-H_2_S by Hcy in macrophages can lead to vascular inflammation.

I/R can reduce the expression of CBS and increase the level of Hcy in renal tissues, thus contributing to the development of renal injuries. CBS can also catalyze the reaction between Hcy and cysteine to generate H_2_S, a molecule playing an essential role in a wide range of pathological and physiological activities. In addition, the administration of NaHS, which is a donor of H_2_S, can improve impaired renal functions in I/R animals. In summary, these findings suggested that the production of H_2_S in tissues can protect the kidney against I/R-induced injuries.

RETRACTED

As a type of derivative from adenosine, IFC-305 was demonstrated to reduce the level of COL1A1 via alternating the status of COL1A1 promoter methylation. In addition, IFC-305 treatment can also alter the epigenetic promoter modification of COL1A1 and Pparg genes [9]. Homocysteine is elevated, while the production of H_2_S is reduced in the development of renal I/R [10,11]. The elevated level of homocysteine suppressed the production of H_2_S via epigenetically regulating the expression of CSE [12]. Interestingly, IFC-305, an adenosine derivative, has been shown to modify the methylation status of various genes [9]. In this study, we hypothesized that IFC-305 could participate in the process of H_2_S production, potentially via regulating the promoter methylation of CSE, attenuating renal ischemia-reperfusion injury by promoting the production of H2S via suppressing the promoter methylation of CSE. We therefore probed the effect of IFC-305 on the methylation of CSE promoter and the production of H_2_S in cellular and animal models of renal I/R.

## Materials and methods

### Animal and treatment

In this study, SD rats (male rats, with an average body weight of about 275 ± 25 g) were acquired from our experimental animal center and were then randomly grouped into 4 groups, i.e., a Control group, an IFC group, an I/R group, as well as an I/R + IFC group. The rats in the I/R groups were treated to establish the I/R rat model, while the rats in the IFC-305 groups were treated with 50 mg/kg weight of IFC-305 as described below.

To establish a rat model of I/R injury, renal I/R operation was carried out to all rats in the I/R groups as follows: First, the rats were placed under anesthesia via an intraperitoneal injection of 50 mg/kg body weight of pentobarbital sodium. In the next step, as the body temperature of the rats was maintained at 37 ± 0.5°C using a heat blanket, the renal artery of the left kidney was clamped for 45 ± 15 min using a clamp (Fine Scientific Tools, Vancouver, Canada) according to a procedure described previously (28). After the ischemia procedure was completed, reperfusion of the kidney was carried out immediately and lasted for about 1 h. At the end of the experiment, both kidneys of each rat were collected and placed into a potassium phosphate buffer and stored at 4 C. At the same time, peripheral blood samples were collected from each rat and centrifuged for 15 min at 3,500 *g* and 4°C to separate the plasma fraction, which was used in subsequent analyses of target gene expression. The rats in the IFC-305 groups were treated with 50 mg/kg weight of IFC-305 via intraperitoneal injection for a total of 5 weeks, and the frequency of intraperitoneal injection of IFC-305 was three times per week [13]. IFC-305 was the aspartate salt of adenosine (Cat.no: 58–61-7, Jiangsu Huayu Chemical Co Ltd., Jiangsu, China) prepared with adenosine-free base and L-aspartic acid. After the treatment with IFC-305, the rats were sacrificed and subjected to the same procedures described above for I/R rats. The rats in the Control group underwent the same procedures as those in the I/R groups except for the actual step of I/R induction. All animal experiments were approved by the Animal Ethics Committee of Dongguan People’s Hospital affiliated to Southern Medical University (ID: ART-2019-31).

RETRACTED

### Cell culture and cell transfection

HK-2 cells, a proximal tubular cell line, which is derived from a normal human adult male kidney, were acquired from ATCC and maintained in an F12 medium (Gibco, Thermo Fisher Scientific, Waltham, MA) supplemented with necessary antibiotics and 10% of fetal bovine serum. In all cell culture experiments, the cell culture conditions were 5% CO2 and saturated humidity in a 37°C incubator. When the HK-2 cells reached a level of confluence of about 70%, the cells were randomly divided into 4 groups, i.e., 1. Untreated group; 2. IFC-305 group; 3. 100 uM Hcy group; and 4. 100 uM Hcy + IFC-305 group. HK-2 cells in Hcy and IFC-305 groups were treated with specified concentrations of Hcy or IFC-305 (both from Sigma Aldrich, St Louis, MO) alone or the combination of the two for 48 h before the cells were harvested for subsequent analysis.

### Bisulfite sequencing

The status of DNA methylation in the CSE promoter of renal tissue in different groups of rats was analyzed using bisulfite sequencing PCR, which was carried out by utilizing a CpGenome DNA bisulfite sequencing PCR assay kit (Serologicals, Norcross, GA) in accordance with the standard protocol provided by the manufacturer.

### Assay of lipid peroxidation

The lipid peroxidation levels in the renal tissues collected from the rats of different groups were measured via determining the levels of MDA using a TBARS assay kit (Sigma Aldrich, St. Louis, MO) in accordance with the standard protocol provided by the manufacturer.

### Assay of superoxide anion

The superoxide anion levels in the renal tissues collected from the rats of different groups were measured using a commercially available superoxide anion assay kit (Sigma Aldrich, St. Louis, MO) in accordance with the standard protocol provided by the manufacturer.

### Measurement of plasma H_2_S

The levels of H_2_S in the plasma samples collected from the rats of different groups were measured using a commercially available Radiello™ Hydrogen Sulfide Starter Kit (Sigma Aldrich, St. Louis, MO) in accordance with the standard protocol provided by the manufacturer.

RETRACTED

### Measurement of plasma creatinine

The levels of creatinine in the plasma samples collected from the rats of different groups were measured via utilizing a commercially available assay kit (Wako Chemical Industries, Mountain View, CA) in accordance with the standard protocol provided by the manufacturer.

### RNA isolation and real-time PCR

Collected tissue and cell samples were initially homogenized in a 4 C PBS buffer (Gibco, Thermo Fisher Scientific, Waltham, MA) placed on ice. Then, the content of total RNA in each sample was isolated by using an RNeasy mini assay kit (Promega, Madison, WI) in accordance with the standard protocol provided by the manufacturer. In the next step, the isolated RNA in each sample was subjected to reverse transcription carried out using a GoScript™ Reverse Transcription Assay Kit (Promega, Madison, WI) in accordance with the standard protocol provided by the manufacturer. Then, the expression level of CSE mRNA in each sample was assayed using real-time PCR carried out on an MX3005P Real-Time PCR machine (Stratagene, San Diego, CA) by using an SYBR Green Master Mix (ABI, Foster City, CA). The assay system and conditions of real-time PCR were prepared in accordance with the standard protocol provided by the manufacturer. Finally, the level of relative expression of CSE mRNA in each sample was calculated using the threshold values obtained from real-time PCR amplifications. The forward primer used for CSE mRNA quantification was 5'- GAACGGCTCTTTACTATGCGAGG-3', and the reverse primer used for CSE mRNA quantification was 5'-CTGAAGAGCCAGGAAGTGTGAG-3'. The relative expression of CSE mRNA was normalized to the expression of GAPDH mRNA. The forward primer of GAPDH mRNA was 5'-GTCTCCTCTGACTTCAACAGCG-3', and the reverse primer of GAPDH mRNA was 5'-ACCACCCTGTTGCTGTAGCCAA-3'.

### Western blot analysis

Western blot analysis was carried out to determine the protein expression of CSE in collected tissue and cell samples. In brief, all samples were lysed in a Radio Immunoprecipitation Assay (RIPA) lysis buffer system (Sangon, Shanghai, China) in accordance with the standard protocol provided by the manufacturer. Then, the content of total proteins in each sample was isolated by centrifuging the lysate for 30 min at 15,000 *g* and 4°C to collect the supernatant. After the protein concentration in each supernatant sample was quantified by using a BCA Assay Kit (Sangon, Shanghai, China), the protein in each sample was resolved via using 10% SDS-PAGE and then blotted onto a PVDF membrane, which was successively incubated with anti-CSE primary antibodies and appropriate HRP-conjugated secondary IgG antibodies (both from Abcam, Cambridge, MA). Finally, the protein bands of each sample were visualized via using a kit of enhanced chemiluminescence reagent (Forevergen, Guangzhou, China) to calculate the relative protein expression of CSE in each sample.

RETRACTED

### Hematoxylin and eosin stain (H&E) staining

H&E staining was carried out to detect the morphology of renal tissues collected from the rats of different groups using a commercially available H&E staining assay kit (Sigma Aldrich, St. Louis, MO) in accordance with the standard protocol provided by the manufacturer.

### ELISA

To measure the activity of CSE, H_2_S, MDA, and superoxide in renal tissue samples and peripheral blood samples collected from the rats of different groups, various commercially available ELISA assay kits (Abcam, Cambridge, MA) were utilized in accordance with the standard protocol provided by the kit manufacturer. Then, the activity of CSE, H_2_S, MDA, and superoxide in each sample was calculated based on its OD value of absorbance measured on an SMR multimode plate reader (Uscn Kit, Wuhan, China).

### Statistical analysis

SPSS version 21.0 (SPSS Inc, Chicago, IL) was utilized for all data analysis. Continuous data showing a Gaussian distribution was displayed as mean ± standard deviations (Mean ± SD). The comparisons of the differences between two groups were evaluated using Student’s *t*-tests, while the comparisons of the differences among multiple groups were evaluated using one-way analysis of variance (ANOVA). The level of statistical significance was determined by *P*< 0.05.

## Results

### IFC-305 treatment prevented I/R induced kidney injury

In this study, we aimed to study the effect of IFC-305 in the treatment of renal I/R injury. We hypothesized that IFC-305 could participate in the process of H_2_S production, potentially via regulating the promoter methylation of CSE, attenuating renal ischemia-reperfusion injury by promoting the production of H2S via suppressing the promoter methylation of CSE. Rats were purchased for this study and then grouped into four groups: Control group, IFC group, I/R group, and I/R + IFC group. An I/R (ischemia/reperfusion) rat model was established and then treated with IFC-305. H&E staining was performed to evaluate the extent of kidney injury in different groups. The kidney injury of I/R rats was significantly increased, while the IFC-305 treatment effectively alleviated the extent of I/R-induced kidney injury (Figure 1(a)). Furthermore, the level of creatinine was measured to evaluate the renal function in the four groups. The creatinine level was remarkably higher in I/R rats but was reduced to a certain degree by the IFC-305 treatment (Figure 1(b)).

RETRACTED

**Figure 1.** IFC-305 treatment prevented I/R induced kidney injury (* P value < 0.05, vs control group; # P value < 0.05, vs. I/R group). A: H&E staining showed an increased level of renal injury in I/R rats, while the IFC-305 treatment alleviated the severity of I/R-induced renal injury (magnification, x200; arrow denotes injured renal tubules). B: The level of creatinine was increased in I/R rats and reduced by IFC-305 treatment.

### Up-regulation of Hcy and down-regulation of CSE in the renal tissue and blood of I/R rats

The concentration of Hcy (homocysteine) in renal tissues (Figure 2(a)) and peripheral blood (Figure 2(b)) was analyzed to show that the Hcy concentration in I/R rats was notably elevated, while the treatment with IFC-305 effectively reduced the Hcy concentration in I/R rats. Since CSE plays a crucial role in regulating Hcy metabolism in the kidney, the CSE activity was measured by ELISA (Figure 2(c)). And the expression of CSE mRNA and protein were, respectively, measured by PCR (Figure 2(d)) and Western blot (Figure 2(e)). All the above results showed that I/R rats had apparently inhibited CSE, while the treatment with IFC-305 recovered CSE to a certain degree.

**Figure 2.** Up-regulation of Hcy and down-regulation of CSE in the renal tissue and blood of I/R rats (* P value < 0.05, vs Control group; # P value < 0.05, vs. I/R group). A: Hcy concentration was elevated in the renal tissue of I/R rats and suppressed by subsequent IFC-305 treatment. B: Hcy concentration was elevated in the peripheral blood of I/R rats and suppressed by subsequent IFC-305 treatment. C: ELISA analysis showed that the decreased CSE activity in the renal tissue of I/R rat was restored by IFC-305 treatment. D: qPCR analysis showed that the decreased CSE mRNA expression in the renal tissue of I/R rat was restored by IFC-305 treatment. E: Western blot analysis showed that the decreased CSE protein expression in the renal tissue of I/R rat was restored by IFC-305 treatment.

### IFC-305 restored the normal DNA methylation status of the CSE promoter in I/R rats

DNA methylation is one of the most important epigenetic factors affecting gene expression. In this study, bisulfite sequencing PCR was performed to analyze the status of DNA methylation in the CSE promoter of renal tissue in different groups of rats. The level of DNA methylation of the CSE promoter was dramatically increased in the renal tissue of I/R rats, while the treatment with IFC-305 effectively reduced the DNA methylation of the CSE promoter (Figure 3).

RETRACTED

**Figure 3.** IFC-305 reduced the abnormally high level of DNA methylation of the CSE promoter in the renal tissue of I/R rats. The level of DNA methylation of CSE promoter was enhanced in the renal tissue of I/R rats and repressed by subsequent IFC-305 treatment.

### The administration of IFC-305 restored the normal levels of H_2_S, MDA and superoxide in the renal tissue and peripheral blood of I/R rats

H_2_S concentration was obviously reduced in the renal tissue (Figure 4(a)) and peripheral blood (Figure 4(b)) of I/R rats, while the administration with IFC-305 remarkably increased the H_2_S concentration. On the contrary, the levels of MDA (Figure 4(c)) and superoxide (Figure 4(d)) were significantly up-regulated in the renal tissue of I/R rats, while the administration of IFC-305 apparently reduced the levels of MDA and superoxide.

**Figure 4.** IFC-305 restored the normal levels of H_2_S, MDA and superoxide in the renal tissue and peripheral blood of I/R rats (* P value < 0.05, vs Control group; # P value < 0.05, vs. I/R group). A: H_2_S concentration was decreased in the renal tissue of I/R rats and restored by subsequent IFC-305 treatment. B: H_2_S concentration was decreased in the peripheral blood of I/R rats and restored by subsequent IFC-305 treatment.C: MDA was increased in the renal tissue of I/R rats and reduced by subsequent IFC-305 treatment. D: Superoxide was increased in the renal tissue of I/R rats and reduced by subsequent IFC-305 treatment.

### IFC-305 increased the activity of CSE in HK-2 cells

One hundred uM of Hcy were added to HK-2 cells to establish a cellular model of I/R. ELISA was then used to measure the activity of CSE in HK-2 cells cultured under different conditions: 1. Untreated, 2. IFC-305, 3. Hcy (100 uM), and 4. Hcy (100 uM) + IFC-305. The Hcy treatment substantially suppressed the CSE activity in HK-2 cells, while the treatment with IFC-305 restored the CSE activity to a certain degree (Figure 5(a)). Similarly, qPCR (Figure 5(b)) and Western blot (Figure 5(c)) analyses showed that Hcy-induced inhibition of CSE mRNA and protein expression was rescued by IFC-305 treatment. In addition, the DNA methylation of the CSE promoter was dramatically increased by Hcy treatment in HK-2 cells, while the treatment with IFC-305 remarkably reduced the level of CSE promoter methylation in HK-2 cells (Figure 6).

**Figure 5.** IFC-305 restored the normal CSE activity in HK-2 cells undergoing Hcy treatment (* P value < 0.05, vs. untreated group; # P value < 0.05, vs. Hcy group). A: ELISA analysis showed that the decreased CSE activity in HK-2 cells undergoing Hcy treatment was restored by the subsequent IFC-305 treatment. B: qPCR analysis showed that the decreased CSE mRNA expression in the HK-2 cells undergoing Hcy treatment was restored by the subsequent IFC-305 treatment. C: Western blot analysis showed that the decreased CSE protein expression in the HK-2 cells undergoing Hcy treatment was restored by the subsequent IFC-305 treatment.

RETRACTED

**Figure 6.** IFC-305 reduced the abnormally high level of DNA methylation of CSE promoter in Hcy-treated HK-2 cells. The level of DNA methylation of CSE promoter was enhanced in Hcy-treated HK-2 cells and repressed by subsequent IFC-305 treatment.

### IFC-305 restored the normal levels of H_2_S, MDA and superoxide in the HK-2 cells treated with Hcy

The treatment of HK-2 cells with Hcy substantially decreased H_2_S concentration, while the treatment with IFC-305 remarkably elevated the H_2_S concentration in supernatant (Figure 7(a)) and cells (Figure 7(b)). On the other hand, Hcy substantially elevated the levels of MDA and superoxide in HK-2 cells, while the treatment with IFC-305 remarkably reduced the levels of MDA (Figure 7(c)) and superoxide (Figure 7(d)) in HK-2 cells.

**Figure 7.** IFC-305 restored the normal levels of H_2_S, MDA and superoxide in Hcy-treated HK-2 cells (* P value < 0.05, vs. untreated group; # P value < 0.05, vs. Hcy group). A: H_2_S concentration was decreased in the supernatant of Hcy-treated HK-2 cells and restored by IFC-305 treatment. B: H_2_S concentration was decreased in Hcy-treated HK-2 cells and restored by IFC-305 treatment. C: MDA was increased in Hcy-treated HK-2 cells and reduced by IFC-305 treatment. D: Superoxide was increased in Hcy-treated HK-2 cells and reduced by IFC-305 treatment.

## Discussion

Renal I/R injuries can occur during the process of renal transplantation as well as the operation of renal resection. Currently, renal I/R injuries are a major contributor of acute renal failures. In addition, I/R can disrupt the metabolism of Hcy in renal tissues, causing the accumulation of Hcy as well as the increased levels of oxidative stress and apoptosis [14]. Hcy is generated in the metabolism process of methionine. In a recent paper, Bearden and his colleagues demonstrated that the delivery of extracellular Hcy can reduce the level of oxidative stress in endothelial cells [15].

Hcy can be produced via the metabolism of methionine. Subsequently, Hcy turns into cysteine under the actions of CSE as well as CBS. As a result, the restriction in methionine intake can reduce the expression of CBS as well as the level of H_2_S [16]. Although the mechanisms involved in the regulation of CSE transcription remain largely unknown, it is suspected the presence of DNA methylation can affect the expression level of its host genes. Indeed, it was shown previously that the increased level of DNA methylation in the promoter of the CSC gene can be triggered by the treatment with Hcy. In this study, we established rat and cellular models of I/R and treated them with IFC-305 to evaluate the therapeutic effect of IFC-305 on I/R-induced renal injury. In addition, we performed H&E staining to evaluate the extent of renal injury of different groups of rats. The results showed that the extent of renal injury was significantly increased in I/R rats, while the IFC-305 treatment efficiently alleviated the extent of renal injury. Furthermore, we carried out ELISA, qPCR and Western blot assays to assess the activity of CSE in the renal tissue of rats and HK-2 cells receiving different treatments. The activity of CSE was apparently decreased in I/R rats and cells, while the treatment with IFC-305 restored the activity of CSE.

RETRACTED

As an H_2_S precursor, Hcy is converted to H_2_S via the catalysis occurring under the action of CSE and CBS. In addition, CSE activity can be inhibited by Hcy to block the synthesis of H_2_S in macrophages, and the presence of DNA methyltransferase (DNMT) can enhance the activity of Hcy.

As a critical enzyme participating in the conversion of methionine into cysteine, CSE was demonstrated to rely on a sufficient cysteine supply to produce glutathione, which acts as a key anti-oxidant in cells.

As a signal transmitter playing a myo-relaxant role in cells, H_2_S is primarily generated by L-cysteine under the catalytic actions of CBS as well as CSE. In fact, both CSE and CBS can participate in the conversion of L-Cys to H_2_S in the uterus tissues of mice. In addition, similar to other signal transmitters such as carbon monoxide and NO, H_2_S can be synthesized endogenously from L-Cysteine under the actions of CBS as well as CSE [17,18]. In this study, we used bisulfite sequencing PCR to analyze the level of DNA methylation in the CSE promoter in I/R rats and cells. The level of DNA methylation was dramatically elevated in I/R models, while the IFC-305 treatment efficiently reduced the level of DNA methylation. In addition, we examined the levels of H_2_S, MDA and superoxide in I/R rats and cells. The results showed that the level of H_2_S was reduced in I/R rats and cells, while the IFC-305 treatment rescued the normal level of H_2_S. In addition, the levels of MDA and superoxide were elevated in I/R rats and cells, while the IFC-305 treatment reduced the levels of MDA and superoxide.

H_2_S is a well-known and important regulator in maintaining the function of both the cardiovascular and the nervous systems [19]. Indeed, it was demonstrated recently that, as a neuro-protective agent, H_2_S at its physiological concentration can inhibit the proliferation of smooth muscle cells by activating the MAPK-signaling pathway while protecting pancreatic cells, cardiomyocytes, neurons, as well as vascular smooth muscle cells against various types of oxidative stress [20–24]. In particular, the I/R of the kidney can trigger the peroxidation of lipids as well as the apoptosis of renal cells. When the synthesis of H_2_S is reduced, the extent of renal injuries can become more severe as manifested by increased levels of lipid peroxidation as well as enhanced cell apoptosis.

RETRACTED

It was suspected that the onset of I/R injuries during kidney transplantation leads to graft dysfunction in about one-third of the cases [25]. Interestingly, I/R can cause elevated oxidative stress and the activation of NF-B, as well as the infiltration of macrophages into renal tissues [26].

Both CGL and CBS can induce the synthesis of H_2_S, which is then involved in the regulation of renal functions [27]. In case of I/R induced renal injury, the synthesis of H_2_S has declined. However, CBS seems to be resistant to I/R-induced changes, thus playing an essential role in maintaining the expression levels of H_2_S in renal tissues.

## Conclusion

In summary, the findings of this study demonstrated that in I/R rats and cells, the level of Hcy was elevated, while the production of H_2_S was reduced by enhancing the methylation of CSE promoter. Furthermore, IFC-305, an adenosine derivative, was able to modify the methylation status of CSE promoter to promote the production of H_2_S and subsequently attenuate the extent of renal injury.

## Data Availability

The data that support the findings of this study are available from the corresponding author upon reasonable request.
